# FK506 binding protein 10: a key actor of collagen crosslinking in clear cell renal cell carcinoma

**DOI:** 10.18632/aging.203359

**Published:** 2021-08-13

**Authors:** Yubai Zhang, Yue Yin, Sijia Liu, Lei Yang, Changhua Sun, Ruihua An

**Affiliations:** 1 Department of Urology Surgery, The First Affiliated Hospital of Harbin Medical University, Harbin, China; 2 Department of Oncology Radiotherapy, The Second Affiliated Hospital of Harbin Medical University, Harbin, China; 3 Department of Gynecological Radiotherapy, The Affiliated Tumor Hospital of Harbin Medical University, Harbin, China; 4 Department of Urology Surgery, The First Hospital of Harbin, Harbin, China

**Keywords:** FKBP10, clear cell renal cell carcinoma, collagen synthesis, prognosis

## Abstract

Clear cell renal cell carcinoma (ccRCC) is the most common type of malignant tumor in the kidney. With numbers of patients whose physical condition or tumor stage not suitable for radical surgery, they only have a narrow choice of using VEGF/mTOR targeted drugs to control their tumors, but ccRCC often shows resistance to these drugs. Therefore, identifying a new therapeutic target is of urgent necessity. In this study, for the first time, we concluded from bioinformatics analyses and *in vitro* research that FK506 binding protein 10 (FKBP10), together with its molecular partner Lysyl hydroxylase 2 (LH2/PLOD2), participate in the process of type I collagen synthesis in ccRCC via regulating crosslinking of pro-collagen chains. Our findings may provide a potential therapeutic target to treat ccRCC in the future.

## INTRODUCTION

Clear cell renal cell carcinoma (ccRCC) is the most lethal cancer in the urinary system [1]. Characterized by an asymptomatic disease course, the disease is often diagnosed late and survival prognosis is often poor [2]. According to investigations, males are almost 2 times vulnerable than females [3]. Due to lacking of biomarkers in the early diagnosis of renal cancer, nearly 20–30% of patients have found distant metastasis at the time of diagnosis [4]. Moreover, numbers of patients whose physical condition not suitable for radical surgery or with late-stage tumors have a narrow choice of using VEGF (vascular endothelial growth factor) or mTOR (target of rapamycin) targeted drugs to control their tumors. Although the development and application of VEGF/mTOR targeted drugs have extended the survival period of many patients, however, these existing targeted drugs often fail to show satisfactory efficacy because of drug resistance. In this circumstance, such patients must undergo cycles of drug resistance and finally be sensitive to no drug. Thus, identifying a new therapeutic target for ccRCC patients is of urgent necessity.

As the most abundant component of extracellular matrix (ECM), collagen has been found not only to be a physical barrier but also involved in tumor infiltration, angiogenesis, invasion, and migration [5]. The aberrantly regulated collagen is found in cancer at the levels of expression, modification, deposition, and degradation [6]. Of all the processes of collagen synthesis, crosslinking is a key step for pro-collagen chains to assemble into collagen triple helix. It has been reported that massive synthesis, thickening, and linear crosslinking facilitates metastasis of tumor cells [7].

FK506 binding protein 10 (FKBP10) and its collaborative protein lysyl hydroxylase 2 (LH2/PLOD2) are the most critical molecules in this collagen crosslinking process. FKBP10 is the gene that encodes the highly conserved 65-kDa protein FK506 binding protein (FKBP65). FKBPs are identified as chaperones and as peptidylprolyl isomerase (PPIase) involved in protein conformation folding during the process of protein transportation and secretion [8]. FKBP10 mainly localizes in the endoplasmic reticulum (ER). In ER, FKBP10 forms a complex with PLOD2, and promotes PLOD2 dimerization, which is crucial for PLOD2 enzymatic activity to hydroxylate Lys residues in the telopeptides of pro-collagen chains [9]. Defect of FKBP10 in fetus leads to collagen synthesis failure and therefore renders a congenital disease named Bruck Syndrome which is characterized by bone fragility and recurring bone fractures [10].

Recent studies revealed that FKBP10 was actively involved in cancers. Giorgio et al. reported that FKBP10 was negatively correlated with the survival of lung cancer patients [11], a similar result was also reported in gastric cancer [12]. A single *in vitro* study also found FKBP10 regulates cell cycle progression and invasion of ccRCC cell line [13]. However, the exact mechanism of FKBP10 in ccRCC remains unclear, its role in collagen synthesis and cancer cell proliferation needs to be elucidated.

In this study, we conclude that FKBP10, together with its collaborative protein PLOD2, are high expressed in ccRCC, and the two genes are negatively correlated with patients’ survival. FKBP10 is involved in the process of collagen biosynthesis in ccRCC cell line. Down-regulation of FKBP10 induces ER stress in ccRCC cell line. Based on the results, we further hypothesize that FKBP10 influences proliferation of ccRCC, reduced collagen crosslinking induced by targeted down-regulation of FKBP10 may sensitize ccRCC to adjuvant therapies.

## RESULTS

### The difference of FKBP10, PLOD2 and pro-collagen I chains in ccRCC and normal kidney tissues

We compared transcriptional levels of FKBP10, PLOD2 and pro-collagen I chains in cancer tissues with normal samples by inquiring ONCOMINE database [14]. The mRNA expression level of FKBP10, PLOD2 and pro-collagen I chains was significantly upregulated in patients with ccRCC. In Gumz’s dataset [15], FKBP10 and PLOD2 were overexpressed compared with that in normal samples with a fold change of 13.212 and 4.249, both rank top 2% of over-expression genes (Figure 1A, 1B). For mRNA expression level of pro-collagen I chains in Gumz’s dataset, Collagen Type I Alpha 1 Chain (COL1A1) and Collagen Type I Alpha 2 Chain (COL1A2) showed fold changes of 3.850 and 9.055 respectively (Figure 1C, 1D). Indicating that not only mRNA of FKBP10 and PLOD2 but also pro-collagen I chains were aberrantly over-expressed.

**Figure 1:** **FKBP10, PLOD2 and pro-collagen I shows high transcription level in ccRCC.** Levels of FKBP10, PLOD2 and pro-collagen I mRNA were significantly higher in ccRCC than in normal tissue. Fold change, associated *p* values, and overexpression gene rank are shown. (**A**) FKBP10 mRNA expression level in Gumz Renal dataset. FKBP10 presented a fold change of 13.212, ranking top 2% in overexpression gene. (**B**) PLOD2 mRNA expression level in Gumz Renal dataset. PLOD2 presented a fold change of 4.249, ranking top 2% in overexpression gene. (**C**), (**D**) COL1A1 and COL1A2 mRNA expression level in Gumz Renal dataset. COL1A1 and COL1A2 presented a fold change of 3.850 and 9.055 respectively, both ranking top 2% in overexpression gene.

### FKBP10 and PLOD2 are strongly stained in IHC analysis

As shown in Figure 2, IHC data obtained from the public database HPA [16] gave us a direct visual result that FBP10 and PLOD2 displayed a strongly stained pattern in ccRCC tissues (Figure 2A, 2B), in contrast, normal kidney tissues have a relatively low level of FKBP10 and PLOD2 (Figure 2C, 2D).

**Figure 2:** **Immunohistochemistry analysis of FKBP10 and PLOD2 in ccRCC. Immunohistochemistry data of FKBP10 and PLOD2 in ccRCC samples and normal kidney tissues from the HPA database.** (**A**) FKBP10 in normal kidney tissue. Antibody HPA057021, patient ID 1859. FKBP10 in glomeruli: staining not detected, weak intensity, quantity<25%, located in cytoplasmic/membranous; FKBP10 tubules: low staining, weak intensity, quantity 25%-75%, membranous. (**B**) PLOD 2 in normal kidney tissue. Antibody CAB025898, patient ID 1933. PLOD2 in glomeruli: low staining, moderate intensity, quantity<25%, located in cytoplasmic membranous; PLOD2 tubules: medium staining, moderate intensity, quantity>75%, membranous. (**C**) FKBP 10 in ccRCC tissue. Antibody HPA057021, patient ID 3039. FKBP10 in ccRCC tissue: high staining, strong intensity, quantity>75%, located in cytoplasmic/membranous. (**D**) PLOD2 in ccRCC tissue. Antibody CAB025898, patient ID 2564. PLOD2 in ccRCC tissue: high staining, strong intensity, quantity>75%, located in cytoplasmic/membranous.

### The prognostic values of FKBP10 in ccRCC

Next, we investigated prognosis data of FKBP10 and PLOD2 in ccRCC patients. Kaplan-Meier plotter [17] was employed in this section. As shown in Figure 3A and 3B, the Kaplan-Meier plotter calculated that higher mRNA expression of FKBP10 and PLOD2 were significantly associated with poor ccRCC patients’ Overall Survival (OS). Further survival analysis of different gender subgroups using UALCAN showed that regardless of different gender, patients with higher FKBP10 and PLOD2 mRNA expression levels presented shorter OS than those with lower levels (Figure 3C and 3D).

**Figure 3:** **High FKBP10 and PLOD2 level predicts poor prognosis in ccRCC patients.** The prognostic value of FKBP10 and PLOD2 level in ccRCC patients. High expression groups has lower survival probability than low expression groups for both genes. (**A**) Effect of FKBP10 expression level on ccRCC patients’ OS. Logrank *p* = 6.6e-10, HR = 2.51. (**B**) Effect of PLOD2 expression level on ccRCC patients’ OS. Logrank *p* = 1.8e-06, HR = 2.06. (**C**) Effect of FKBP10 expression level and gender on ccRCC patients’ OS. Logrank *p* = 0.0021. (**D**) Effect of PLOD2 expression level and gender on ccRCC patients’ OS. Logrank *p* = 0.00052.

### Gene correlation network and protein-protein interaction network of FKBP10

Top 50 positive genes correlated with FKBP10 and PLOD2 analyzed by LinkedOmics were presented as heatmaps. Both analyses of FKBP10 and PLOD2 share each other in top50 positively correlated genes (Figure 4A and 4B).

**Figure 4:** **Genes correlated with FKBP10 and PLOD2 in ccRCC, and PPI network of FKBP10.** (**A**) Heat map showing top50 genes positively correlated with FKBP10 in ccRCC, PLOD2 was ranked. (**B**) Heat map showing top50 genes positively correlated with PLOD2 in ccRCC, FKBP10 was ranked. (**C**) PPI network of FKBP10 analyzed by String database. PLOD2, COL1A1 and COL1A2 showed strong interaction with FKBP10 (interaction score > 0.7).

To explore the biological function partners of FKBP10, we used String to construct and analyze the protein-protein interaction (PPI) network via public database String [18]. The result indicates that PLOD2, COL1A1, COL1A2 list among the top 10 proteins which interact with FKBP10 (genes combined score > 0.7) (Figure 4C).

### Gene ontology analysis reveals that FKBP10 mainly involves in collagen synthesis in ccRCC

We then performed gene ontology analysis of FKBP10 and its correlated genes analyzed by String (FKBP10, LEPRE1, KDELR3, CRTAP, SERPINH1, PPIB, COL1A1, PLOD2, TMEM38B, GTF2IRD1, COL1A2) using the g:GOSt Functional profiling tab of g:Profiler [19]. The functional profiling results reported that the functional roles of the target gene list focus mainly on the aspect of collagen synthesis. The genes in the list are involved in Molecular Function: collagen binding (GO:0005518), extracellular matrix structural constituent conferring tensile strength (GO:0030020), cis-trans isomerase activity (GO:0016859) (Figure 5A); Biological Process: collagen fibril organization (GO:0030199), extracellular matrix organization (GO:0030198), peptidyl-proline modification (GO:0018208), peptidyl-lysine hydroxylation (GO:0017185), collagen metabolic process (GO:0032963) (Figure 5B); Cellular Component: endoplasmic reticulum lumen (GO:0005788), endoplasmic reticulum (GO:0005783), collagen type I trimer (G:0005584), collagen trimer (GO:0005581), fibrillar collagen trimer (GO:0005583), banded collagen fibril (GO:0098643), complex of collagen trimers (GO:0098644) (Figure 5C).

**Figure 5:** **Gene Ontology analysis reports FKBP10 and its correlated genes are densely involved in collagen synthesis.** (**A**) Molecular function analysis of FKBP10 in ccRCC: collagen binding (GO:0005518), extracellular matrix structural constituent conferring tensile strength (GO:0030020), cis-trans isomerase activity (GO:0016859). (**B**) Biological process analysis of FKBP10 in ccRCC: collagen fibril organization (GO:0030199), extracellular matrix organization (GO:0030198), peptidyl-proline modification (GO:0018208), peptidyl-lysine hydroxylation (GO:0017185), collagen metabolic process (GO:0032963). (**C**) Cellular component analysis of FKBP10 in ccRCC:: endoplasmic reticulum lumen (GO:0005788), endoplasmic reticulum (GO:0005783), collagen type I trimer (G:0005584), collagen trimer (GO:0005581), fibrillar collagen trimer (GO:0005583), banded collagen fibril (GO:0098643), complex of collagen trimers (GO:0098644).

### FKBP10 is high expressed in ccRCC cell lines

We next performed western blot in ccRCC cell line 786-O. Normal kidney cell line HK2 was set as control. In consistent with the bioinformatics result, western blot result revealed that FKBP10 was high expressed in ccRCC cell line 786-O, whereas normal kidney cell line HK2 presented a low FKBP10 expression pattern (Figure 6A).

**Figure 6:** **FKBP10 is high expressed and its inhibition causes ER stress in ccRCC.** β-actin is set as loading control. Quantitative analysis of each study is presented in a bar graph. (**A**) Immunoblotting showed FKBP10 was high expressed in 786-O ccRCC cell line comparing with normal kidney HK-2 cell line. (**B**) FKBP10 RNAi efficacy was confirmed by immunoblotting. (**C**) After FKBP10 RNAi, ER stress marker CHOP was high expressed than negative control group. (**D**) After FKBP10 RNAi, collagen type I precursor COL1A1 aberrantly accumulated in ccRCC cells. Negative control group showed much less expression of COL1A1.

### Down-regulation of FKBP10 brings about the rise in ER stress

48 hours after RNAi transfection (Figure 6B), ccRCC cell line 786-O transfected with FKBP10 interference RNA was tested for pro-collagen I expression and ER stress. Not surprisingly, interference of FKBP10 deranged crosslinking of collagen type-I, causing pro-collagen I accumulation (Figure 6C). The accumulation of the pro-collagen brought about overexpression of ER stress marker CHOP (Figure 6D).

## DISCUSSION

Our study identified FKBP10 as a promising therapeutic target in ccRCC based on bioinformatics analyses by inquiring various public databases and *in vitro* research. Initially, we found FKBP10 and its molecular partner PLOD2, together with their potential substrate COL1A1 and COL1A2 presented a high-expression profile in ccRCC patients using a database that analyzes GEO datasets. To achieve a direct visual comprehension of FKBP10 and PLOD2 protein levels in ccRCC, IHC data from the HPA database were employed. IHC data were consistent with mRNA expression data that ccRCC expressed high level of FKBP10 and PLOD2. Besides, patients with higher FKBP10 and PLOD2 levels inclined to have poorer OS and RFS than the ones with lower expression. No obvious OS differences were observed between different genders, indicating that FKBP10 has the potential to be a therapeutic target for all genders. Biological function analyses revealed FKBP10 and its correlated genes participate in various biological processes and pathways, especially in the processes related to collagen modification, indicating FKBP10 did actively participate in collagen synthesis in ccRCC. Finally, *in vitro* experiments verified that FKBP10 was aberrantly high expressed in ccRCC cell lines and a following RNA interference of FKBP10 presented accumulation of pro-collagen I and rise in ER stress.

Being the most abundant component of the extracellular matrix, collagens act more as a progression facilitator for malignant tumors than just a protective physical barrier. As reported, collagen gets involved in linearized deposition, hypoxia response, tumor angiogenesis, tension derived epithelial–mesenchymal transition of malignant tumor [7]. Almost all these processes require remodeling or rearranging of collagen fibers, which relies on frequent crosslinking and re-crosslinking of collagen chains.

FKBP10 was first thought to be involved in diseases such as idiopathic pulmonary fibrosis [20] and osteogenesis imperfecta [21]. Interestingly, almost all previous studies proved that FKBP10 was greatly involved in collagen synthesis. In recent years, researchers turn to elucidate its role in cancers such as gastric cancer [12], prostate cancer [22], and ovarian cancer [23]. Ge et al. even gave a glimpse into the phenotype effect of FKBP10 in ccRCC at cell line level and a small number of samples [13]. Most cancers just mentioned presented an FKBP10 positively correlated behavior, i.e., high expression level of FKBP10 promotes cancer and predicts poor prognosis [12, 13, 22, 24].

Here we postulate a mechanism that FKBP10, together with its collaborative molecule PLOD2, are engaged in the process of massively synthesizing and secreting type I collagen from ER in ccRCC. FKBP10-dependent PLOD2 dimer stabilization may be indispensable for type I collagen crosslinking [9]. Telopeptide lysyl hydroxylation mediated by FKBP10 and PLOD2 is critically important for proper crosslinking and polymerization of collagen I fibrils [25]. This high activity leads to dynamical homeostasis in the process of protein precursors folding into correct conformation. Once this fragile homeostasis gets imbalanced, such as FKBP10 mutates defectively or being inhibited by targeted drugs, un-crosslinked pro-collagen I will accumulate. These accumulated protein precursors brought about high ER stress.

ER stress emerges as a novel cancer treatment mechanism in the recent decade based on the theory that cells tend to undergo apoptosis when ER proteins, including FKBP10, fail to correctly fold protein precursors to be synthesized afterwards [26] such as pro-collagen. It has been proved by a study that pro-collagen I appeared to aggregate in FKBP10 null cells, then ER stress induced by pro-collagen I bursts [21, 27]. Under this stressed circumstance, cells tend to proceed apoptosis [28].

In conclusion, we analyzed the expression and prognostic value of FKBP10 in ccRCC in this study. Our results indicate that FKBP10 and its collaborative molecule PLOD2 are involved in crosslinking of type I collagen in ccRCC. Silencing of FKBP10 interrupts the crosslinking and brings about high ER stress. With the ER-stressed apoptotic tending status, cancer cell may be vulnerable to physio-chemical environment changes, such as ionizing radiation beam, chemical therapy drugs or radiofrequency ablation. The high FKBP10 expression could also serve as a prognosis predictor. Furthermore, FKBP10 may be a candidate therapeutic target for ccRCC patients or other cancer types with high FKBP10 level.

## MATERIALS AND METHODS

### ONCOMINE analysis

ONCOMINE (https://www.oncomine.org), an online cancer microarray database, was used to analyze the transcription level of FKBP10 in ccRCC. The mRNA expression of FKBP10, PLOD2, COL1A1 and COL1A2 in clinical cancer samples were compared with that in normal people, using a Students’ *t*-test to generate a *p*-value. The cut-off of *p*-value and fold change were set as 0.01 and 1.5, respectively.

### UALCAN analysis

UALCAN (http://ualcan.path.uab.edu/) was used to analyze the survival possibility of different gender subgroups. UALCAN uses TCGA level 3 RNA-seq and clinical data from 31 cancer types, providing an interactive website to perform in-depth analyses of TCGA gene expression data. The site allows analysis across various tumor subgroups based on individual cancer stages, tumor grade, genders or other clinicopathological features.

### HPA analysis

HPA (https://www.proteinatlas.org/) database was used to obtain immunohistochemistry data in ccRCC patients and normal kidney tissues. The HPA database stocks transcriptome and proteome data generated from RNA sequencing analysis and immunohistochemistry analysis.

### Kaplan-Meier plotter analysis

Kaplan-Meier Plotter (http://kmplot.com/analysis/) was used to predict survival situation correlated to FKBP10 and PLOD2 expression. This online database contains gene expression data and survival information of 530 clinical ccRCC patients. To analyze the overall survival (OS), relapse-free survival (RFS), patients were divided into two groups by median expression (high vs. low expression) and assessed by a Kaplan-Meier survival plot, with the hazard ratio (HR).

### LinkedOmics analysis

The LinkedOmics database (http://www.linkedomics.org) is a web-based platform for analyzing 32 TCGA cancer-associated multi-dimensional datasets. LinkedOmics was used to study genes differentially expressed in correlation with FKBP10 and PLOD2 in TCGA ccRCC data (*n* = 533). Results were analyzed statistically using the Pearson correlation test. All results were graphically graphed in volcano plots and heat maps.

### String analysis

String (https://string-db.org/) To further investigate the biological function of FKBP10 in ccRCC, we analyzed the possible interactions of FKBP10 using a protein-protein interaction (PPI) network. An interaction score of 0.7 was set as a cut-off value.

### g:Profiler analysis

g:Profiler (https://biit.cs.ut.ee/gprofiler/) is an online analysis server for functional interpretation of gene lists. g:GOSt tab performs functional enrichment analysis on input gene list. It maps genes to known functional information sources and detects statistically significantly enriched terms.

### Cell culture

Proximal tubular cell line HK-2 (ATCC No. CRL-2190) and ccRCC cell line 786-O (ATCC No. CRL-1932) were obtained from ATCC. Cells were cultured in RPMI-1640 medium (ThermoFisher) supplemented with 10% fetal bovine serum and 1% penicillin/streptomycin at 37°C in humidified air with 5% CO2.

### Reagents

Monoclonal mouse anti-FKBP10 antibody (sc-135907), monoclonal mouse anti-actin antibody (sc-8432), monoclonal mouse anti-CHOP antibody (sc-7351), monoclonal mouse anti-COL1A1 antibody (sc-293182) was purchased from Santa Cruz. HRP conjugated mouse IgG kappa binding protein (sc-516102) was also purchased from Santa Cruz.

### Immunoblotting

786-O and HK-2 cells were prepared into cell extracts for SDS-PAGE and then separated using Mini-PROTEAN System (Bio-Rad). Separated proteins were transferred to PVDF membrane (Immobilon-E PVDF Membrane, 0.45 μm, Merck Millipore) using Mini Trans-Blot Cell (Bio-Rad). After blocking (PBS-T with 3% skimmed milk) for 1 hour at room temperature, primary antibody was incubated overnight at 4°C (1:1000 for sc-135907, sc-8432, sc-7351 and sc-293182; 1:10000 for sc-516102. Then the membranes were washed in blocking buffer and then incubated for secondary antibody probing (1:5000) for 1 hour at room temperature. The blots were detected by Amersham ECL Prime Western Blotting Detection Reagent (RPN2232, GE Healthcare) by using ChemiDoc MP Imaging System (Bio-Rad).

### RNAi and transfection

FKBP10 siRNA (sc-75019) were supplied by SantaCruz. 786-O cell was transfected with FKBP10 siRNA using Lipofectamine™ RNAiMAX Transfection Reagent (Thermo Fisher Scientific) following the manufacturer’s experiment protocol. Validity verification and further experiment was performed 48 hours after transfection.
